# Baicalein Reduces the Invasion of Glioma Cells via Reducing the Activity of p38 Signaling Pathway

**DOI:** 10.1371/journal.pone.0090318

**Published:** 2014-02-28

**Authors:** Zhenni Zhang, Jianrui Lv, Xiaoming Lei, Siyuan Li, Yong Zhang, Lihua Meng, Rongliang Xue, Zongfang Li

**Affiliations:** 1 Anesthesia Department, the Second Affiliated Hospital, School of Medicine, Xi'an Jiaotong University, Xi'an, P. R. China; 2 National-Local Joint Engineering Research Center of Biodiagnostics & Biotherapy, Xi'an Jiaotong University, Xi'an, P. R. China; 3 Key Laboratory of Environment and Genes Related to Diseases of the Education Ministry, School of Medicine, Xi'an Jiaotong University, Xi'an, P. R. China; 4 General Surgeon Department of Cadre's Ward, the Second Affiliated Hospital, School of Medicine, Xi'an Jiaotong University, Xi'an, P. R. China; Duke University Medical Center, United States of America

## Abstract

Baicalein, one of the major flavonids in *Scutellaria baicalensis*, has historically been used in anti-inflammatory and anti-cancer therapies. However, the anti-metastatic effect and related mechanism(s) in glioma are still unclear. In this study, we thus utilized glioma cell lines U87MG and U251MG to explore the effect of baicalein. We found that administration of baicalein significantly inhibited migration and invasion of glioma cells. In addition, after treating with baicalein for 24 h, there was a decrease in the levels of matrix metalloproteinase-2 (MMP-2) and MMP-9 expression as well as proteinase activity in glioma cells. Conversely, the expression of tissue inhibitor of metalloproteinase-1 (TIMP-1) and TIMP-2 was increased in a dose-dependent manner. Moreover, baicalein treatment significantly decreased the phosphorylated level of p38, but not ERK1/2, JNK1/2 and PI3K/Akt. Combined treatment with a p38 inhibitor (SB203580) and baicalein resulted in the synergistic reduction of MMP-2 and MMP-9 expression and then increase of TIMP-1 and TIMP-2 expression; and the invasive capabilities of U87MG cells were also inhibited. However, p38 chemical activator (anisomycin) could block these effects produced by baicalein, suggesting baicalein directly downregulate the p38 signaling pathway. In conclusion, baicalein inhibits glioma cells invasion and metastasis by reducing cell motility and migration via suppression of p38 signaling pathway, suggesting that baicalein is a potential therapeutic agent for glioma.

## Introduction

Malignant glioma, with the invasive and infiltrative character, can constitute up to 10% of tumors in the central nervous system (CNS) [1], and is the leading cause of brain tumor-related death in both developed and developing countries [2]. The most common and aggressive subtype is, classified grade IV astrocytic tumor, the glioblastoma (GBM) [3]. It is characterized by a high proliferation rate and invasiveness, which make it refractory to treatment of local irradiation, surgical extirpation, as well as conventional chemotherapy with temozolomide (TMZ) [4], [5]. According to recent statistics, the average lifespan expectancy of patients with GBM is still less than 14 months, despite several advances achieved currently in multimodal treatments [6].

The extracellular matrix (ECM) affects the biological behavior of both normal and neoplastic cells in several ways, including the regulation of cell attachments, and the motility and invasion of epithelial cells during embryogenesis, organogenesis, tumor development, and metastasis [7]. The breakdown of the ECM is mediated by matrix metalloproteinases (MMPs), particularly MMP-2 and MMP-9, which play important roles in degrading basement membranes and cancer invasion and metastasis [8], [9]. TIMPs are the endogenous inhibitors of the zinc-dependent endopeptidases of the matrix metalloproteinase families [10], [11], [12]. Thus, the degree of ECM breakdown is controlled by the temporal release of MMPs and their inhibition by TIMPs.

MAPKs are serine/threonine protein kinases that participate in intracellular signaling during proliferation, differentiation, cellular stress responses, and apoptosis [13]. The MAPK signaling plays a critical role in the outcome and the sensitivity to anticancer therapies. It has been reported that invasion and metastasis of glioma cells required specific intracellular signaling cascade activations, among which the p38 signaling pathway is considered crucial [14], [15], [16], [17].

Baicalein (5, 6, 7-trihydroxy-2-phenyl-4H-1-benzopyran-4-one) is one of the major flavonids with a defined chemical structure (**Figure 1**) in *Scutellaria baicalensis* that has long been widely used for thousands of years in oriental medicine. Several biological effects of baicalein such as anti-viral, anti-hepatotoxicity, anti-inflammation, and anti-tumor properties have been reported [18], [19], [20]. However, the anti-metastatic effect and related mechanism(s) in glioma cells have not previously been determined. In this study, we tested the hypothesis that administration of baicalein may inhibit the proliferation, migration and invasion of human glioma U87 cells via p38 signaling pathway *in vitro*.

**Figure 1:** Chemical structure of baicalein.

## Materials and Methods

### Reagents

Fetal bovine serum (FBS), penicillin and streptomycin were ordered from Gibco. Baicalein, SB203580 and anisomycin were ordered from Sigma. Dulbecco's modified Eagle's medium (DMEM) was purchased from Invitrogen. Anti-p38, anti-Phospho-p38 (Thr180/Tyr182), anti-MMP-2, anti-MMP-9, anti-TIMP-1 and anti-TIMP-2 antibodies were purchased from Cell Signaling. Anti-β-actin was purchased from Santa Cruz.

### Cell culture

The human glioma cell line U87MG and U251MG (obtained from a cell bank at the Fourth Military Medical University, China) were cultured in DMEM supplemented with 10% FBS, 100 U/ml penicillin and 100 µg/ml streptomycin. All cells were incubated at 37°C with 5% CO_2_.

### Cell viability assays

Cell survival was assessed using standard 3-(4, 5-dimethylthiazol-2-yl)-2, 5- diphenyltetrazolium bromide (MTT) assay in accordance with previously described protocols [21]. Briefly, cells were seeded in 96-well culture plates (2×10^4^ cells per well). The cells were treated with serially diluted concentrations of baicalein. Control wells received culture medium. After 24 h incubation, the cells were washed twice with PBS and incubated with 5 mg/ml MTT (Sigma) for 4 h. The solution was discarded after 2 h (37°C) and 100 µl DMSO was added to each well. The optical density was measured in a microplate reader at 562 nm formazane absorbance.

### *In vitro* invasion and migration assays

The *in vitro* invasion and migration activity was measured according to the methods described previously [22], [23]. Cells were pretreated with 0, 10, 20 and 40 µM baicalein or SB203580 (20 µM) or anisomycin (5 µM/L) for 24 h, surviving cells were harvested and seeded to Boyden chamber (Neuro Probe, Cabin John, MD, USA) at 10^4^ cells/well in serum free medium and then incubated for 24 h at 37°C. For invasion assay, 20 µl Matrigel (25 µg/50 µl; BD Biosciences, MA, USA) was applied to 8 mm pore size polycarbonate membrane filters and the bottom chamber contained standard medium. Filters were then air-dried for 5 h in a laminar flow hood. At the endpoint, the cells on the upper side of inserts were completely removed by swabbing, while the cells on the bottom side of the filter were fixed, stained and counted. The migration assay was carried out as described in the invasion assay with no coating of Matrigel [24], [25].

### Quantitative real-time PCR

Total RNAs were prepared by using the RNeasy Mini kit (Invitrogen). cDNA was synthesized with SuperScript III Reverse Transcriptase (Invitrogen). Real-time quantitative PCR was performed using SYBR Green II in accordance with the PrimeScript RT-PCR Kit protocol (TaKaRa). Gene-specific primer pairs used for amplification were as follows: for β-actin, CCATCGTCCACCGCAAAT (forward) and CATGCCAATCTCATCTTGTTT (reverse); for MMP-2, CTCATCGCAGATGCCTGGAA (forward) and TTCAGGTAATAGGCACCCTTGAAGA (reverse); for MMP-9, GTCCACCCTTGTGCTCTTCC (forward) and GCCACCCGAGTGTAACCAT (reverse). β-actin was used as an endogenous control. The analysis of the relative gene copy number data for MMP-2 and MMP-9 was performed using the comparative 2^−ΔΔCt^ method and were normalized by β-actin in each sample.

### Gelatin zymography

The cells were treated with different concentrations of baicalein or SB203580 at 37°C for 24 h, and samples of conditioned media were collected. Briefly, the conditioned medium was adjusted to the same quantity of total protein (5 mg per load), then treated with SDS-PAGE non-reducing sample buffer without boiling. Samples were separated by 0.1% gelatin-8% SDS-PAGE electrophoresis. Afterwards, the gels were soaked twice in 2.5% Triton X-100 for 30 min for three times at room temperature, and incubated in reaction buffer (10 mM CaCl_2_, 40 mM Tris-HCl and 0.01% NaN_3_, pH 8.0) at 37°C for 12 h. Gels were rinsed with distilled water, stained with Coomassie brilliant blue R-250. The gelatinolytic activities were densitometrically quantified and analyzed by an image analysis system (Bio-Rad Laboratories, Richmond, CA).

### Western blotting analysis

Cells were suspended in lysis buffer (40 mmol/l Tris-HCl, 1 mmol/l EDTA, 150 mmol/l KCl, 100 mmol/l NaVO_3_, 1% Triton X-100, 1 mmol/l PMSF, pH 7.5), after treatment with different concentrations of baicalein,SB203580 or anisomycin, respectively. The proteins were separated by 10% SDS-polyacrylamide gel electrophoresis and transferred onto PVDF membranes. The membranes were subsequently blocked in defatted milk (5% in Tris-buffered saline with TWEEN-20 (TBST) buffer) at room temperature for 1 h to block non-specific binding and were then incubated overnight with antibodies against p38, p-p38, MMP-2, MMP-9, TIMP-1, TIMP-2, ERK1/2, p-ERK1/2, Akt, p-Akt, JNK1/2, p-JNK1/2 or β-actin in TBST containing 5% defatted milk at 4°C. The membranes were then incubated with a HRP goat anti-mouse or anti-rabbit IgG antibody for 1 h at room temperature. The bands were detected with an enhanced chemiluminescence kit (Amersham, ECL Plus, Freiburg, Germany) and exposed by autoradiography. The densitometric analysis was performed using Image J software (GEhealthcare, Buckinghamshire, UK), and the results were expressed as arbitrary units (a.u.).

### Statistical analysis

Experiments were repeated three times, and the results of the studies were expressed as the means ± standard deviation (SD). Statistical differences were analyzed by one-way or two-way ANOVA and further by posthoc tests using the statistical software of GraphPad Prism 5. All statistical tests and corresponding *p*-values were two sided. *p*<0.05 was regarded as significant. We performed correlation analysis by the Z-test.

## Results

### Baicalein inhibits the proliferation of glioblastoma cells

The anti-proliferation effects of baicalein at various concentrations (0 to 60 µM) on U87MG cells are shown in **Figure 2**. At 50 µM, baicalein obviously inhibited the proliferation of U87MG cells, while, at concentrations below 50 µM,the inhibition was not so significant; hence we chose a concentration range of baicalein lower than this for all subsequent experiments.

**Figure 2:** Effect of baicalein on the proliferation of U87MG cells. Cell viability was measured by MTT assay. Values represent the means ± SD of three independent experiments performed in triplicate. *p<0.05 and **p<0.01 compared with the control group.

### Baicalein inhibits the migration and invasion of glioblastoma cells

**Figures 3** shows the effect of baicalein on cell migration and invasion in U87MG cells that were treated with 0, 10, 20 and 40 µM of baicalein for 16 h (cell migration) and 24 h (cell invasion), respectively. Using a cell migration and invasion assay with a Boyden chamber, we showed that baicalein reduced the invasion and migration of U87MG cells substantially in a concentration-dependent manner. Quantification analysis indicated that the inhibition rate of migration and invasion were approximately 25.7%, 58.3%, 76.7% and 41.1%, 65.0%, 80.4%, respectively. Similar anti-metastatic effect of baicalein was observed in U251MG glioblastoma cells (dates shown in **Figure S1**).

**Figure 3:** Effect of baicalein on the migration and invasion of U87MG cells. (A) U87MG cells were pretreated with 0, 10, 20 and 40 µM baicalein for 24 h and then seeded in the upper wells without coating of Matrigel. FBS (10%) was added to the bottom chambers for 16 h to induce cell migration. After 16 h, cells on the bottom side of the filter were fixed, stained and counted. (B) The migration rate was expressed as a percentage of the control (0 µM). (C) U87MG cells were pretreated with 0, 10, 20 and 40 µM baicalein for 24 h and then seeded in the upper wells. FBS (10%) was added to the bottom chambers for 24 h to induce cell invasion. After 24 h, cells on the bottom side of the filter were fixed, stained and counted. (D) The invasion rate was expressed as a percentage of the control (0 µM). Values represent the means ± SD of three independent experiments performed in triplicate. *p<0.05 and **p<0.01 compared with the control group.

### Inhibition effect of baicalein on the transcriptional levels of MMP-2 and MMP-9

We used real-time quantitative PCR (RT-PCR) to investigate the inhibitory effect of baicalein on MMP-2 and MMP-9 in U87MG cells. U87MG cells were treated with 0, 10, 20 and 40 µM baicalein for 24 h and then subjected to RT-PCR. We found that baicalein could significantly reduce the transcriptional levels of MMP-2 and MMP-9 in a concentration-dependent manner (**Figure 4A**). The inhibition rate of MMP-2 was approximately 32.9%, 67.5% and 81.6% after 24 h of treatment with 10, 20 and 40 µM baicalein, while, the MMP-9 was approximately 24.58%, 61.50% and 88.83%, respectively.

**Figure 4:** Baicalein suppresses the expression and activity of MMP-2 and MMP-9 and promotes the expression of TIMP-1 and TIMP-2 in U87MG cells. (A) The effects of baicalein on the expression of MMP-2 and MMP-9 were assessed by RT-PCR. (B) The protein levels of MMP-2 and MMP-9 were analyzed in U87MG cells treated with baicalein (0, 10, 20 and 40 µM) for 24 h using Western blotting. (C) Quantification of (B). (D) Effects of baicalein on the activities of MMP-2 and MMP-9. (E) Quantification of (D). (F) The protein levels of TIMP-1 and TIMP-2 were analyzed in U87MG cells treated with baicalein (0, 10, 20 and 40 µM) for 24 h using Western blotting. (G) Quantification of (F). Values represent the means ± SD of three independent experiments performed in triplicate. *p<0.05 and **p<0.01 compared with the control group.

### Baicalein suppresses the expression and activity of MMP-2 and MMP-9

The expression and activity of MMP-2 and MMP-9 in U87MG cells that were exposed to different concentrations of baicalein were examined, because both MMPs are crucial to cell invasion. Cells were treated with 0, 10, 20 and 40 µM baicalein for 24 h and then subjected to Western blotting. **Figure 4B and 4C** show that baicalein significantly reduces the protein levels of MMP-2 and MMP-9 in a concentration-dependent manner compared with the control group. Gelatin zymography was performed to assess the activity of MMP-2 and MMP-9 in cells treated with various concentrations of baicalein. As shown by gelatinolytic activity data, baicalein inhibited the activity of MMP-2 and MMP-9 in a concentration-dependent manner (**Figure 4D**). Quantification analysis indicated that MMP-2 activity was reduced by 51.6%, 88.6% and 98.5%, and MMP-9 activity by 22.0%, 57.9% and 91.4% in cells that were treated with 10, 20, and 40 µM of baicalein, respectively (**Figure 4E**).

### Baicalein promotes the expression of TIMP-1 and TIMP-2 in U87MG cells

Imbalances between MMPs and TIMPs play important roles in glioma progression and metastasis [26], [27]; thus, the protein level of TIMP-1 and TIMP-2 in U87MG cells was assessed. U87MG cells were treated with 0, 10, 20 and 40 µM baicalein for 24 h and then subjected to Western blotting. **Figure 4F and 4G** showed that baicalein significantly up-regulated the protein levels of TIMP-1 and TIMP-2 in a concentration-dependent manner.

### The p38 signaling pathway is involved in the anti-metastatic mechanism of baicalein

In human glioma cells, activation of p38 signaling pathway is required for the invasion process [28]. Moreover, the mechanism is correlated with proteinases and their inhibitors [29], [30]; thus, the effect of baicalein on the p38 signaling pathway in U87MG cells was investigated. We found that baicalein could reduce the phosphorylation of p38 in a concentration-dependent manner (**Figure 5A and 5B**), but not ERK1/2, JNK1/2 and PI3K/Akt (**Figure S2**).

**Figure 5:** Effect of baicalein on the p38 signaling pathway. (A) The protein levels of p38 and p-p38. (B) Phosphorylation density of p38 was digitally scanned. Values represent the means ± SD of three independent experiments performed in triplicate. *p<0.05 and **p<0.01 compared with the control group.

In order to research whether the inhibitory effect of baicalein on cell invasion and MMP-2 and MMP-9 expression was correlated with inhibition of the p38 signaling pathway, U87MG cells were pretreated with a p38 inhibitor (SB203580, 20 µM) for 30 min and then incubated in the presence or absence of baicalein (10 µM) for 24 h. The results show that treatment with SB203580 and baicalein significantly inhibited cell invasion (**Figure 6A and 6B**) and reduced MMP-2 and MMP-9 protein expression (**Figure 6C and 6D**). Meanwhile, the expression of TIMP-1 and TIMP-2 were increased (**Figure 6C and 6D**). Furthermore, chemical anisomycin, a p38 activator, were used to confirm the role of p38 signaling pathway. As shown in **Figure S3**, anisomycin activated p38 MAPK and could block these effects produced by baicalein, suggesting baicalein directly downregulate the p38 signaling pathway. These results reveal that the inhibition of both cell invasion and MMP-2 and MMP-9 expression by baicalein occurs through the suppression of p38 signaling pathway.

**Figure 6:** Effects of the p38 inhibitor (SB203580) and baicalein on cell invasion and MMP-2, MMP-9, TIMP-1 and TIMP-2 expression in U87MG cells. (A) Cells were pretreated with SB203580 (20 µM) for 30 min and then incubated in the presence or absence of baicalein (10 µM) for 24 h. Cellular invasiveness was measured using the Boyden chamber invasion assay. (B) The percent invasion rate was expressed as a percentage of control. (C, D) The protein levels of MMP-2, MMP-9, TIMP-1 and TIMP-2 were analyzed in treated U87MG cells by Western blotting. Values represent the means ± SD of three independent experiments performed in triplicate. *p<0.05 and **p<0.01 compared with the control group.

## Discussion

Glioma, especially GBM with high morbidity and mortality, is still a serious public health problem around the world [29], and as a administration of the anti-tumor natural products baicalein has been confirmed in many cancers [31], [32], [33], [34]. Up to now, the anti-metastatic effect of baicalein and related mechanism(s) in glioma cells are not clear. In the present study, we investigated whether baicalein could inhibit the invasive and metastatic ability of U87MG cells *in vitro* by regulating of the MMP/TIMP ratio via inhibition of the p38 signaling pathway.

Metastasis is one of the leading causes of cancer-related death among glioma patients. Degradation of the ECM of blood or lymph vessels is critical to metastasis, because loss of the ECM allows cancer cells to invade the blood or lymphatic system and spread to other tissues and organs. MMPs, especially MMP-2 and MMP-9, play critical roles in the degradation of type IV collagen, a major constituent of the ECM, and are closely related to the invasion and metastasis of various cancer cells [22], [35], [36], [37]. Additionally, baicalein has been reported to cause down-regulation of MMP-2 and MMP-9 expression in HCC metastasis [38]. MMP activities can be restrained by TIMPs to prevent extensive ECM degradation. Wang et al. showed that chrysanthemum indicum ethanolic extract (CIE) substantially suppressed the proliferation and invasiveness of a HCC cell line (MHCC97H), with a notable decrease in MMP-2 and MMP-9 expression and a simultaneous increase in TIMP-1 and TIMP-2 expression [34]. In the present study, we found that baicalein suppressed the expression and activity of MMP-2 and MMP-9 and simultaneously promoted TIMP-1 and TIMP-2 expression in glioma cells; thus, the MMP/TIMP balance was restored. These results indicated that the anti-metastatic effect of baicalein on glioblastoma cells was correlated with modulation of MMPs and their inhibitors (TIMPs).

The synthesis of proteinases and their inhibitors are regulated by multiple signaling cascades, including the p38 signaling pathway as well as ERK1/2, FAK, IKK, NF-kappaB-mediated pathways [25], [34], [39]. p38 signaling pathway is widely expressed in various tissues and has much broader functions physiologically [29]. The role of p38 in cancer is disputable, and appears to be influenced by several factors, such as cell type, the extent of activation, etc [40]. The p38 signaling pathway can induce the expression of MMPs and thereby promotes the degradation of ECM proteins, which leads to cell invasion [41]. To further explore the possible mechanism(s) of baicalein in the inhibition of glioma invasion, we have detected the levels of phosphorylation of p38 in U87MG cells. The results demonstrated that the phosphorylation of p38 in cells treated with baicalein was significantly reduced relative to that in control cells, whereas there were no significant changes in the activity of ERK1/2, JNK1/2 and PI3K/Akt signaling pathways. Baicalein combined with a p38 inhibitor (SB203580) significantly reduced glioblastoma cell invasion and was accompanied by downregulation of MMP-2 and MMP-9 and upregulation of TIMP-1 and TIMP-2. However, p38 chemical activator (anisomycin) could block these effects produced by baicalein, suggesting baicalein directly downregulate the p38 signaling pathway.

In conclusion, this study demonstrated the inhibitory effect of baicalein on the invasive and metastatic capability of glioblastoma cells. Furthermore, the downregulation of MMP-2 and MMP-9 induced by baicalein is attributed to suppression of the p38 signaling pathway, which in turn leads to invasion and metastasis of glioblastoma cells by baicalein. These findings reveal a new potential therapeutic application of baicalein in anti-metastatic therapy for glioma.

## Supporting Information

Figure S1 **Effect of baicalein on the migration and invasion of U251MG cells.** (A) U251MG cells were pretreated with 0, 10, 20 and 40 µM baicalein for 24 h and then seeded in the upper wells. FBS (10%) was added to the bottom chambers for 24 h to induce cell invasion. After 24 h, cells on the bottom side of the filter were fixed, stained and counted. (B) The invasion rate was expressed as a percentage of the control (0 µM). Values represent the means ± SD of three independent experiments performed in triplicate. *p<0.05 and **p<0.01 compared with the control group.
(TIF)

Figure S2 **Effect of baicalein on ERK1/2, JNK1/2 and PI3K/Akt signaling pathways.** (A) The protein levels of ERK1/2 and p-ERK1/2. (B) Phosphorylation density of ERK1/2 was digitally scanned. (C) The protein levels of AKT and p-AKT. (D) Phosphorylation density of AKT was digitally scanned. (E) The protein levels of JNK1/2 and p-JNK1/2. (F) Phosphorylation density of JNK1/2 was digitally scanned.
(TIF)

Figure S3 **Effects of the p38 activator (anisomycin) and baicalein on cell invasion.** (A) After treating with anisomycin (25 µg/ml) for 30 min, the expression of p38 and p-p38 was detected. (B) Cells were pretreated with anisomycin (25 µg/ml) for 30 min and then incubated in the presence or absence of baicalein (40 µM) for 24 h. Cellular invasiveness was measured using the Boyden chamber invasion assay. (C) The percent invasion rate was expressed as a percentage of control. (D) The inhibition rates of baicalein on two groups of cells. Values represent the means ± SD of three independent experiments performed in triplicate. *p<0.05 and **p<0.01 compared with the control group.
(TIF)
